# Baicalein restrains proliferation, migration, and invasion of human malignant melanoma cells by down-regulating colon cancer associated transcript-1

This article has been retracted.

**DOI:** 10.1590/1414-431X20198934

**Published:** 2019-11-21

**Authors:** Xiaoliang Yang, Jinjie Jiang, Chunyan Zhang, Yinghao Li

**Affiliations:** 1 Department of Burn and Plastic Surgery, Qingdao Central Hospital, The Affiliated Central Hospital of Qingdao University, Qingdao, Shandong, China; 2 Department of Traditional Chinese Medicine, Qingdao Central Hospital, The Affiliated Central Hospital of Qingdao University, Qingdao, Shandong, China

**Keywords:** Malignant melanoma, Colon cancer associated transcript-1, Wnt/β-catenin, MEK/ERK

## Abstract

Baicalein (BAI) is an acknowledged flavonoids compound, which is regarded as a useful therapeutic pharmaceutical for numerous cancers. However, its involvement in melanoma is largely unknown. This study aimed to examine the anti-melanoma function of BAI and unraveled the regulatory mechanism involved. A375 and SK-MEL-28 were treated with BAI for 24 h. Then, CCK-8 assay, flow cytometry, and transwell assay were carried out to investigate cell growth, migration, and invasion. RT-qPCR was applied to detect the expression of colon cancer associated transcript-1 (CCAT1) in melanoma tissues and cells. The functions of CCAT1 in melanoma cells were also evaluated. Western blot was utilized to appraise Wnt/β-catenin or MEK/ERK pathways. BAI restrained cell proliferation and stimulated cell apoptotic capability of melanoma by suppressing cleaved-caspase-3 and cleaved-PARP. Cell migratory and invasive abilities were restrained by BAI via inhibiting MMP-2 and vimentin. CCAT1 was over-expressed in melanoma tissues and down-regulated by BAI in melanoma cells. Overexpressed CCAT1 reversed the BAI-induced anti-growth, anti-migratory, and anti-invasive effects. Furthermore, BAI inhibited Wnt/β-catenin and MEK/ERK pathways-axis via regulating CCAT1. Our study indicated that BAI blocked Wnt/β-catenin and MEK/ERK pathways via regulating CCAT1, thereby inhibiting melanoma cell proliferation, migration, and invasion.

## Introduction

Melanoma evolves from skin mucosa or pigmented membrane and is the most common cancer with high metastatic potential (1). Malignant melanoma, caused by the abnormal transformation of normal melanocytes, is one of the fastest growing malignant tumors with an annual growth rate of 3–5% (2). To date, surgery and chemotherapy combined with immunotherapy are the most common endorsed therapeutic approaches to melanoma (3,4). Nevertheless, the biggest disadvantage of these therapies is toxicity. Thus, there is research focused on natural products towards cell metastasis of melanoma (5). However, the potential value of traditional Chinese medicine in the treatment of melanoma has not been assessed.

*Scutellaria baicalensis* Georgi is a kind of traditional Chinese medicine containing several flavonoids. One of the ingredients is baicalein (BAI), which is commonly regarded as useful adjuvant therapeutic pharmaceutical for various diseases (6). Thus far, a number of researchers tested the efficacy of BAI on malignant tumors, such as breast carcinoma (7), non-small-cell lung carcinoma (8), cervical carcinoma (9), and carcinoma of urinary bladder (10). Moreover, previous research indicated that BAI impeded cell proliferation and melanogenesis of B16F10 mouse melanoma cells (11,12). What is not yet clear is the functional mechanism of BAI on human malignant melanoma.

Long noncoding RNAs (lncRNAs) are RNA segments with no fewer than 200 nucleotides in length that do not encode proteins (13). lncRNAs are closely linked to miscellaneous regulations, functioning as regulators of gene transcription, RNA splicing, and miRNA regulatory systems (14,15). A number of investigators reported that lncRNAs SLNCR1 and HEIH interfered with the melanoma cell proliferative potential, migratory status, and invasive ability via regulating corresponding downstream targets (16,17). Colon cancer associated transcript-1 (CCAT1), an innovative tumor-related lncRNA, plays an essential role in tumor progression, being up-regulated in malignancies (18). However, the extent to which CCAT1 is related to malignant melanoma remains poorly understood.

Here, we demonstrated a crucial role of BAI in inhibiting cell growth and motility by mediating CCAT1 as well as the underlying mechanism of BAI-induced signaling pathways in human melanoma cells. Our findings might provide new insights into the application of traditional Chinese medicine and feasible therapies for malignant melanoma.

## Material and Methods

### Clinical tissues

Twenty-two pairs of human melanoma tissues and corresponding paracancerous skin specimens were collected from patients at Qingdao Central Hospital (Qingdao, Shandong) from January 2017 to July 2018. Thirteen cases were from males and 9 were from females, who did not receive any radiation or chemotherapy before surgery. Participants signed an authorization and the Ethics Committee of Qingdao Central Hospital approved the procedures and the study.

### Cell culture and treatment

The malignant melanoma cell lines A375 and SK-MEL-28, which were cultured in DMEM (Gibco, USA) enriched with 10% fetal bovine serum (FBS, Gibco), were obtained from ATCC (USA). The conditions for cell culture were 5% CO_2_ and 37°C. BAI was obtained from Nanjing ZeLang Medical Technology Co. Ltd. (#ZL100708, China). BAI was diffused in DMSO as a storage concentration and diluted using DMEM to work concentrations (100, 50, 20, and 10 μM). The cells were treated with BAI for 24 h.

### Cell transfection

The entire length of CCAT1 was concatenated into the pcDNA3.1 vector (GenePharma, China). The recombination plasmid was termed as pCCAT1. The lipofectamine 2000 reagent (Life Technology, USA) was used for the cells transfection. The stably transfected cells were cultured in DMEM combined with 0.5 mg/mL G418 (Solarbio, China). Four weeks later, stable transfected cells were formed.

### Cell viability assay

Cells (5×10^3^/well) were seeded into 96-well plates and were raised for 48 h. After treatment with BAI, 10 μL Cell Counting Kit-8 (CCK-8, Dojindo, USA) solutions were added to the cultures. Then, cultures were incubated for 1 h at 37°C. Microplate Reader (Bio-Rad, USA) was employed to evaluate the cell viability at 450 nm.

### Bromodeoxyuridine (BrdU) assay

Cell proliferation was determined using BrdU (Sigma-Aldrich, USA). After treatment of BAI, BrdU (1 mg/mL) was added to the cells for 3 h. Then, immunofluorescence assay was carried out to estimate the BrdU-tagged cells, providing the cell proliferation rate.

### Cell migration and invasion assays

Cell migratory capacity and invasive potential were assessed by transwell culture chamber (Corning Cosatar, USA), which consists of 8-μm pore polycarbonate membrane. Firstly, 200 μL of 1×10^4^ cells, which were cultured in DMEM without FBS, were seeded into the top chamber, which had been covered with Matrigel matrix (Becton Dickinson, USA) for invasion assay or kept uncovered for migration assay. Consequently, 800 μL medium was injected to the lower chamber. After 24 h, the migratory cells were fixed with methyl alcohol and dyed with 0.5% crystal violet liquid (Solarbio). Then, the relative migration rates were calculated. After 48 h, the invading cells were processed in the above same manner and the number of invading cells was counted.

### Apoptosis assay

Apoptotic cells proportion was measured utilizing PI/FITC-Annexin V staining kit (Invitrogen, USA). In brief, cells (1×10^6^/well) were cultured into 6-well plates and starved in FBS-free medium for 12 h. Next, PI and Annexin V-FITC solutions were added to the cell cultures. Flow cytometry was performed with FACScan (Becton Dickinson). The apoptosis ratio was calculated using FlowJo software (Becton Dickinson).

### Reverse transcription and quantitative real-time PCR (RT-qPCR)

Trizol reagent (Life Technologies Corporation, USA) was utilized to isolate total RNA of tissue samples and cell cultures. Reverse transcription of RNA was implemented utilizing SuperRT cDNA Synthesis Kit (Cwbio, China). SYBR^®^ Green PCR Kit (Qiagen, Germany) was employed for qPCR analysis to detect CCAT1 expression. qPCR was executed on iQ5 real-time PCR Detection system (Bio-Rad). The mRNA expression of CCAT1 was normalized with β-actin. The relative quantification of CCAT1 in tumor tissues and cells was calculated using the equation: amount of target = 2^-ΔΔCt^ (19).

### Western blot

Total proteins were extracted from cells utilizing RIPA lysis buffer (Cwbio), which contains phenylmethylsulfonyl fluoride (PMSF, Solarbio). Proteins were quantified by the Super-Bardford Pritein Assay Kit (Cwbio). The extractions were loaded into 12% polyacrylamide gel on the Bis-Tris Gel system (Bio-Rad). The products were transferred onto polyvinylidene fluoride (PVDF) membranes, which were then cultivated at 4°C overnight with primary antibodies. The primary antibodies included anti-cleaved-caspase-3 (#ab2303, Abcam, USA), anti-cleaved-PARP (#ab3246, Abcam), anti-MMP-2 (#ab37150, Abcam), anti-vimentin (#ab92547, Abcam), anti-Wnt3a (#ab219412, Abcam), anti-β-catenin (#ab32572, Abcam), anti-t-MEK (#9126, Cell Signaling Technology, USA), anti-p-MEK (#9154, Cell Signaling Technology), anti-t-ERK (#9102, Cell Signaling Technology), anti-p-ERK (#4370, Cell Signaling Technology), and anti-β-actin (#ab179467, Abcam). Then, the PVDF membranes were rinsed and incubated with horseradish peroxidase-conjugated goat anti-rabbit IgG (#ab6721, Abcam) and goat anti-mouse IgG (#ab205719, Abcam) for 1 h at 20°C. After washing, the PVDF membranes were treated with ChemiDoc™ XRS system (Bio-Rad), and the intensity of bands was finally evaluated with ImageJ software (NIH, USA).

### Statistical analysis

Each experiment was repeated three times. Graphpad 6.0 software (USA) was utilized for statistical analysis. Data are reported as means±SD. Analysis of variance (ANOVA) and Student's *t*-test were applied to calculate P values. A P value <0.05 was regarded as significant.

## Results

### BAI attenuated cell proliferation and promoted cell apoptosis of malignant melanoma cells

Figure 1A presents the inhibition of BAI on cell viability. Cells were sensitive to 20 μM BAI compared with the untreated group (P<0.01). Cell viability was impeded by BAI with an inhibitory concentration of 50% (50 μM). Therefore, 50 μM was considered to be an acceptable concentration for the next proliferation and apoptosis assay. Figure 1B shows that BAI (50 μM) significantly inhibited the cell proliferation of A375 and SK-MEL-28 cells compared to the untreated cells (P<0.001). Reversely, flow cytometry using PI/FITC-Annexin V indicated that BAI promoted cell apoptosis compared with the untreated group (P<0.01, Figure 1C). We analyzed the expression of cleaved-caspase-3, which acted in cell apoptosis and participated in the cleavage of repair enzymes, such as PARP (20). The protein expression analysis was consistent with the result of flow cytometry. BAI treatment accelerated cleaved-caspase-3 and cleaved-PARP expression compared with the untreated cells (P<0.001, Figure 1D). The experiments detected some evidence for the inhibitory effect of BAI on the growth of malignant melanoma cells.

**Figure 1:** Baicalein (BAI) attenuated cell proliferation and strengthened cell apoptotic capacity of malignant melanoma cells. **A**, Cell viability of A375 and SK-MEL-28 cells followed by 24-h treatment with BAI (0, 10, 20, 50, and 100 μM) was assessed by CCK-8. **B**, Cell proliferation of melanoma cells was examined by bromodeoxyuridine (BrdU) assay. **C**, Flow cytometry was utilized to assess the apoptotic rate of melanoma cells. **D**, Expression of cleaved-caspase-3 and cleaved-PARP was tested by western blot assay. The relative expression of protein was normalized by β-actin. Data are reported as mean±SD. **P<0.01, ***P<0.001 (ANOVA). ns: not significant; CTRL: control.

### BAI inhibited cell migratory capacity and invasive potential of melanoma cells

As indicated in Figure 2A, BAI significantly suppressed cell migration compared to control group (P<0.001). Figure 2B shows the results obtained from the preliminary analysis of Matrigel invasion assay. When melanoma cells were stimulated with BAI, there was an obvious decline in the relative invasive rate compared to the control group (P<0.001). It is well known that the activation of angiogenesis depends on MMP-2 and vimentin, which are known to participate in the epithelial-mesenchymal transition (21,22). As shown in Figure 2C, MMP-2 and vimentin expression was inhibited due to the treatment of BAI compared with the control (P<0.001). Overall, these results indicated that BAI apparently impaired the motility of malignant melanoma cells.

**Figure 2:** Baicalein (BAI) inhibited the cell migratory capacity and invasive potential of melanoma cells. **A**, Migration of A375 and SK-MEL-28 cells, treated or not with BAI, was examined by transwell assay. **B**, Invasion of A375 and SK-MEL-28 cells was detected by transwell assay with Matrigel matrix. **C**, Protein expression of MMP-2 and vimentin was tested by western blot assay. The relative expression of protein was normalized by β-actin. Data are reported as mean±SD. ***P<0.001 (*t*-test). CTRL: control.

### CCAT1 was up-regulated in melanoma tissues and down-regulated by BAI in melanoma cells

As can be seen in Figure 3A, CCAT1 expression was increased in melanoma specimens compared with the non-tumor tissues (P<0.001). Furthermore, BAI-induced down-regulation of CCAT1 (P<0.001) in malignant melanoma cells was also confirmed by RT-qPCR (Figure 3B). Thus, there might be an association between BAI and CCAT1.

**Figure 3:** CCAT1 was up-regulated in melanoma tissues and down-regulated by baicalein (BAI) in melanoma cells. **A**, Expression of CCAT-1 in malignant melanoma tissues (n=22) and non-tumor skin specimens (n=22) was analyzed by RT-qPCR. **B**, Expression of CCAT-1 in malignant melanoma cells after treating with BAI or not was determined by RT-qPCR. Data are reported as mean±SD. ***P<0.001 (*t*-test). CTRL: control.

### BAI inhibited growth of malignant melanoma cells via regulating CCAT1

To better understand the underlying molecular mechanisms, including a possible role for CCAT1, exogenous overexpression of CCAT1 was implemented by transfection of pCCAT1 into A375 and SK-MEL-28 cells (Figure 4A). After stable transfection with plasmid, cells were treated with 50 μM BAI. Proliferation assay showed that BAI suppressed the proliferation capacity of malignant melanoma cells compared to control (P<0.001, Figure 4B). However, the suppression was reversed by the CCAT1 overexpression (P<0.001). In parallel, the promotion of BAI on cell apoptosis was also reduced in A375 and SK-MEL-28 cells. Furthermore, western blot analysis revealed that the protein levels of cleaved-caspase-3 and cleaved-PARP were markedly decreased in response to the combined influence of BAI and CCAT1 (P<0.001, Figure 4D). In summary, above data indicated that BAI inhibited cell growth and promoted cell apoptotic potential via weakening CCAT1.

**Figure 4:** Baicalein (BAI) inhibited the growth of malignant melanoma cells via regulating CCAT1. **A**, RT-qPCR assay was used to estimate CCAT1 expression in A375 and SK-MEL-28 after transfection with pCCAT1. **B** and **C**, BradU assay and flow cytometry assays were utilized to evaluate overexpression of CCAT1 and BAI on cell proliferation and apoptosis. **D**, Western blot assay evaluated the relative expression levels of cleaved-caspase-3 and cleaved-PARP. The relative expression of protein was normalized by β-actin. Data are reported as mean±SD. *P<0.05, ***P<0.001 (ANOVA). CTRL: control.

### BAI suppressed migration and invasion of malignant melanoma via regulating CCAT1

Subsequently, we detected the cell migratory capacity and invasive potential in response to the treatment of BAI and overexpressed CCAT1. Melanoma cells featured a decreased relative migratory rate and invasion rate with BAI treatment compared with the untreated group (P<0.001, Figure 5A,B). We also discovered that the group transfected with pCCAT1 and then treated with BAI exhibited increased cell migration and invasion rate compared to the group transfected with pcDNA3.1 and then treated with BAI (P<0.001). Concomitantly, we examined whether BAI could negatively regulate MMP-2 and vimentin expression through regulating CCAT1. As shown in Figure 5C, the protein expression of MMP-2 and vimentin were remarkably increased in CCAT1 overexpressed cells, which were not treated with BAI. Together, these results demonstrated that BAI exerted its negative function of cell metastasis via regulating CCAT1 expression in malignant melanoma cells.

**Figure 5:** Baicalein (BAI) suppressed the migration and invasion of malignant melanoma via regulating CCAT1. **A** and **B**, Transwell assay was utilized to test the relative cell migratory and invasive rates. **C**, Western blot was utilized to analyze MMP-2 and vimentin expression levels in melanoma cells treated with BAI or BAI+pCCAT1. The relative expression of proteins was normalized by β-actin. Data are reported as mean±SD. *P<0.05, ***P<0.001 (ANOVA). CTRL: control.

### BAI suppressed CCAT1 to block Wnt/β-catenin and MEK/ERK signaling pathway-axis

The well-known tumor factor regulator, CCAT1, has been shown to have an overwhelming association with tumor proliferation and apoptosis by activating Wnt/β-catenin and MEK/ERK signaling pathways (23,24). To address whether the above signaling pathways were involved in the function of BAI, protein expression was detected by western blot. Compared with the untreated group, the protein levels of Wnt3a and β-catenin were decreased in BAI-treated cells and were reversed by exogenous CCAT1 (P<0.001, Figure 6A). Similarly, the protein levels of p-MEK and p-ERK were also suppressed by BAI (P<0.001, Figure 6B). The results indicated that BAI blocked Wnt/β-catenin or MEK/ERK pathways by negatively regulating CCAT1.

**Figure 6:** Baicalein (BAI) suppressed CCAT1 to block Wnt/β-catenin and MEK/ERK signaling pathway. **A**, The expression of Wnt3a and β-catenin and, **B**, of p-MEK, p-ERK, t-MEK, and t-ERK were examined by western blot. The relative expression of proteins was normalized by β-actin. Data are reported as mean±SD. ***P<0.001 (ANOVA). CTRL: control.

## Discussion

Numerous active components extracted from traditional Chinese medicinal plants exert multiple pharmacological effects (25). Among these, perhaps the most unexpected finding was that BAI induced growth of HeLa cells via mitochondrial and death receptor pathways (9). Although it has been reported that BAI could act as an essential anti-tumor modulator, leading to ameliorated biological processes, such as programmed cell death and angiogenesis in the B16F10 cells (26), the underlying molecular mechanisms remained to be fully demonstrated. Our study found that there were intricate regulating effects between BAI and the progression of malignant melanoma.

BAI is a vigorous herbal medicine that exerts indispensable functions towards the cardiovascular system and hepatoma (27,28). The function of BAI mainly displays as two aspects: anti-oxidative and inhibitory action on cell growth. Chou et al. (11) showed that BAI caused a reduction in cellular viability of melanoma cells through generating ROS scavengers. Existing research recognized that BAI inhibited tumor growth via activation of cleaved-caspase-3 (26). The results of our study were in line with the above previous experiments. We found that BAI alleviated cell growth, and migratory and invasive ability in malignant melanoma. Our findings indicated that BAI exerted indispensable functions as tumor suppressor.

It was reported that abnormal expression of lncRNAs might be related to a wide spectrum of tumor biological processes (29). Reports such as that conducted by Wu et al. (30) show that overexpression of CCAT1 significantly elicit cell proliferation and invasion and inhibit cell cycle in clear cell renal cell carcinoma. Beyond that, Lv et al. (31) verified that CCAT1 served as an oncogenic factor in melanoma genesis, accumulating cell proliferation, migration, and invasion abilities. However, there is a relative paucity of literature concerning CCAT1 involvement in regulating the effects of BAI on melanoma biological processes. In this study, we measured CCAT1 expression level and found that CCAT1 was up-regulated in melanoma. We showed for the first time that BAI inhibited cell proliferation, migration, and invasion of malignant melanoma via regulating CCAT1.

Wnt3a is a key activator of Wnt pathway, generally triggering the acknowledged Wnt/β-catenin signaling pathway (32) and is related to diversified biological processes, such as cell growth and migration (33,34). The MAPK/ERK signaling pathway regulates cell proliferation and differentiation in many tumor cells (35,36) and is associated with melanin synthesis (37). Debates have been raised about the signaling pathway involved in the progression of malignant melanoma. Results from earlier studies demonstrated that BAI inhibited melanogenesis through activation of the ERK signaling pathway but did not induce AKT activation (12). Recent investigators found that BAI impeded the migratory and invasive potential of B16F10 cells through the suppression of PI3K /AKT signaling pathway (38). The present experiments uncovered the down-regulated protein expression of Wnt3a, β-catenin, p-MEK, and p-ERK in malignant melanoma cells treated with BAI. The restraint was reversed by exogenous expressed CCAT1. Therefore, we speculated that BAI blocked Wnt/β-catenin or MEK/ERK signaling pathways by regulating CCAT1.

Overall, our study indicated that BAI hindered Wnt/β-catenin and MEK/ERK signaling pathways by regulating CCAT1, thereby inhibiting proliferation, migration, and invasion of melanoma cells. The present study demonstrated a pivotal role of BAI in tumor regulation, which might provide new light on the development of therapeutic strategies against malignant melanoma. Comprehensive *in vivo* experiments are crucial for future research.
